The article "Intervention of Shugan Xiaozhi Decoction on Nonalcoholic Fatty Liver Disease via Mediating Gut-Liver Axis" was published in 2022. Journal: Biomed Res Int.

# Intervention of Shugan Xiaozhi Decoction on Nonalcoholic Fatty Liver Disease via Mediating Gut-Liver Axis

**DOI:** 10.1155/2022/4801695

**Published:** 2022-07-05

**Authors:** Huili Yang, Lian Feng, Linyi Xu, Dansheng Jiang, Fenfen Zhai, Guangdong Tong, Yufeng Xing

**Affiliations:** ^1^Hepatology Department, Shenzhen Traditional Chinese Medicine Hospital, Shenzhen, Guangdong 518033, China; ^2^The Fourth Clinical Medical College of Guangzhou University of Chinese Medicine, Shenzhen, Guangdong 518033, China; ^3^Shenzhen Futian Center for Chronic Disease Control, Shenzhen, Guangdong 518048, China

## Abstract

Nonalcoholic fatty liver disease (NAFLD) is a chronic liver disease with an increasing incidence rate but few therapies. Shugan Xiaozhi decoction (SX) has demonstrated beneficial effects in treating NAFLD with an unclear mechanism. This study was aimed at investigating the therapeutic mechanism of SX on high-fat diet-induced NAFLD rats via the gut-liver axis. Hepatic steatosis and integrity of intestinal mucosa in NAFLD rats were assessed by histopathological staining. The level of lipid and inflammation were estimated by enzyme-linked immunosorbent assay. Western Blotting was used to detect apolipoprotein (apo) B48 expression. 16S rRNA analysis was used to measure the changes of gut microbial composition after SX treatment. The expressions of zona occludens 1 protein (ZO-1), occludin, and secretory immunoglobulin A (sIgA) in the colon were detected by immunostaining to investigate the intestinal barrier function. Our study found that SX reduced hepatic steatosis, the levels of alanine aminotransferase, aspartate aminotransferase, total cholesterol, and triglyceride and apoB48 expression but increased peroxisome proliferator activated receptor *α* (PPAR*α*) level. Moreover, SX altered the diversity of gut microbiota, upregulating the relative abundance of *f_Prevotellaceae*, while downregulating *f_Bacteroidales_ S24-7*, *f_Lachnospiraceae*, *f_Ruminococcaceae*, *f_Erysipelotrichaceae*, and *f_Desulfovibrionaceae*. By increasing the expression of ZO-1 and occludin and decreasing the level of proinflammatory factors, including sIgA, lipopolysaccharide, tumor necrosis factor-*α*, interleukin-1*β*, monocyte chemotactic protein-1, and transforming growth factor-*β*1, SX improved intestinal mucosal integrity and barrier function. Our study illustrated that the gut-liver axis was a potential way for SX to ameliorate NAFLD, that is, by regulating the expression of PPAR*α*, apoB48, and modulating gut microbiota to protect the intestinal barrier function, and thus alleviate lipid deposition and inflammatory response in the liver.

## 1. Introduction

Nonalcoholic fatty liver disease (NAFLD) is common clinicopathological syndrome characterized by fatty degeneration of hepatocytes and lipid accumulation, of which, natural history includes nonalcoholic simple fatty liver (NAFL), nonalcoholic steatohepatitis (NASH), and associated liver cirrhosis and hepatocellular carcinoma (HCC) [1, 2]. As the second most common cause of liver transplantation currently, NAFLD is predicted to be the main indication for liver transplantation and the main reason of liver-related morbidity and mortality, within 20 years [3]. Unfortunately, the morbidity of NAFLD shows a rapid growth and younger trend over recent years. It is estimated that the global prevalence of NAFLD is around 25.24% [4]. At present, the current majority standpoint recognized that the hypothesis of “multiple-hits” could explain the pathogenesis of NAFLD more accurately, which involved factors such as liver fat deposition, insulin resistance (IR), intestinal disorders, lipotoxicity, inflammation, oxidative stress, c-Jun N-terminal kinase signaling, and epigenetic dysregulation [5–7].

Liver lipid metabolism disorder is one of the most common initial inducement of NAFLD and continue to influence the disease progress [8]. Free fatty acids (FFAs) were synthesized by excess dietary fatty acids via de novo lipogenesis (DNL) and continuously produced triglyceride (TG) in the liver, resulting in abnormally elevated level of intrahepatic TG, which could be considered a NAFLD biomarker [9, 10]. Apolipoprotein (apo) B48 is an apolipoprotein synthesized and secreted by the intestine and plays an important role in the control of lipid transport [11]. It has been suggested that defective production and/or secretion of apo B lipoproteins were highly associated with fatty degeneration of the liver and might involve impaired synthesis of very low-density lipoproteins (VLDL), resulting in the accumulation of TG in the liver [12]. In addition, IR, a possible pathogenesis of NAFLD, had positive correlation with the raised plasma levels of apoB48-containing lipoproteins, which might be due to impaired hepatic ability of clearing TG-rich lipoproteins caused by excessive production of intestinal chylomicrons (CMs) and accumulation of serum CM remnants [13, 14]. On the other hand, cholesterol absorption is mainly accomplished by the endocytosis of exogenous cholesterol through peroxisome proliferator activated receptors (PPARs) and low-density lipoprotein receptor (LDL-R), while cholesterol excretion is through the bile acid pathway [15]. PPARs exist in a variety of tissues with active metabolism such as the liver and participate in regulating the absorption and metabolism of cholesterol, phospholipids, and FFAs [16]. PPARs have *α*, *β*, *γ*, and *δ* subtypes, among which, highly expressed PPAR*α* has been recognized to mitigate NAFLD by enhancing lipid metabolism and may affect the editing of apo B mRNA [16, 17].

Studies have shown that intestinal microbiota dysbiosis is one of the key factors of “multiple-hits” and takes a significant role in the progress of NAFLD via the gut-liver axis [18–21]. There are about ten times as many gut microbes as there are cells in the human body, with the dominant flora, *Firmicutes* and *Bacteroidetes*, in the gut [18, 22]. However, the intestinal microbial diversity of NAFLD patients significantly changed, presenting decreased *Bacteroidetes* but increased *Firmicutes* [18]. The imbalance of intestinal microbial composition and abundance would loosen tight junctions and damage the arrangement of nearby intestinal epithelial cells, leading to impaired intestinal barrier function and enhanced intestinal permeability [23]. This disrupted gut barrier allows lipopolysaccharide (LPS) and other intestinal microbial metabolites, to enter the circulation and cause inflammation in the liver [10, 24, 25]. The translocation of LPS could trigger immune response and raise the levels of inflammatory cytokines, such as tumor necrosis factor-*α* (TNF-*α*) and interleukin-1*β* (IL-1*β*) [26]. Besides, the gut microbiota could regulate the lipid metabolism of NAFLD by changing the formation of intestinal lipoproteins and regulating metabolites, such as bile acids and short-chain fatty acids, to affect the absorption and clearance of lipids [27, 28]. Therefore, regulating the intestinal microbiota to ameliorate intestinal permeability, reduce inflammation, and modulate lipid metabolism has been deemed to be an underlying approach to relieve NAFLD [29].

More and more attention has been focused on the effects of traditional Chinese medicine on NAFLD by acting on lipid metabolism and intestinal microbiota [30]. In fact, traditional Chinese medicine can modulate lipid metabolism, increase the abundance of intestinal flora, repair intestinal barrier function, and reduce inflammation, thus improving NAFLD [30]. Our research group has been consistently absorbed in investigating the effect of Shugan Xiaozhi decoction (SX) on NAFLD and has found that it could significantly improve the lipid deposition, but its effect on intestinal microbiota in NAFLD is still unclear [31]. Thus, this study further explored the impact of SX on gut microbiota and the expression of key protein in lipid metabolism PPAR*α* and apoB48 in NAFLD via the gut-liver axis (Figure 1).

## 2. Materials and Methods

### 2.1. Drugs

SX is composed of Artemisiae Scopariae Herba, Nelumbinis folium, Pumex, Cassiae Semen, Crataegi Fructus, Alismatis Rhizoma, Poria, Aurantii Fructus Immaturus, Bupleuri Radix, Gardeniae Fructus, Paeoniae radix alba (stir-baked), and Glycyrrhizae Radix et Rhizoma in a proportion of 6 : 6 : 6 : 6 : 6 : 6 : 4 : 3 : 2 : 2 : 1 : 1. Guangdong Yifang Pharmaceutical Co., Ltd. (China) manufactured and supplied all herbal drugs in formula granules form. Before use, the granule drugs of SX were dissolved and mixed in water.

### 2.2. Animal and Drug Administration

40 male Sprague-Dawley (SD) rats (200 ± 20 g, 8 weeks), provided by the Animal Center of Chengdu University of Traditional Chinese Medicine, were adaptively fed for a week at the animal center with the relative humidity of 40 ± 10%, temperature of 22 ± 3°C, and 12 h light/dark alternation. Water and food are freely available to all animals. The Animal Ethics Committee of Chengdu Dashuo experimental animal Co., Ltd., had reviewed and granted this research (IACUC-20170731024).

After acclimatization, SD rats were randomly divided into the normal group, model group, SX-H group, and SX-L group (*n* = 10). All feed came from Sichuan Provincial Medical Laboratory Animal Center (Sichuan, China). The rats in the normal group were fed with standard chow composed of 76% carbohydrate, 10% fat, and 14% protein, while the other three groups were fed with high-fat diet (HFD) added 10% lard, 10% protein, and 1% cholesterol to the standard feed. According to the equivalent doses of rats and humans calculated by Experimental Methodology of Pharmacology and the results of our early studies [31], the SX-H group and SX-L group were, respectively, treated with 40 and 20 g/kg SX per day. The normal group and model group were given the same amount of normal saline. From the first day of modeling, intragastric administration was performed once a day for 12 weeks. Moreover, rats were weighed once a week to adjust the dose. After treatment, the venous blood, liver, small intestine, and intestinal feces were collected under anesthesia by 3% barbituric acid (Solarbio, Beijing, China) through intraperitoneal injection.

### 2.3. Enzyme-Linked Immunosorbent Assay (ELISA)

At the end of the intervention, a sufficient amount of venous blood and the liver tissue were collected. After anesthetizing the rats, blood was collected from the portal vein through a syringe. The blood was centrifuged at 1,000xg/min for 10 min to separate and collect serum and plasma which were, respectively, used to measure the content of alanine aminotransferase (ALT), aspartate aminotransferase (AST), total cholesterol (TC), and TG and the level of LPS. The liver tissues were cleaned with precooled PBS, then placed in a glass homogenizer, and added with precooled PBS for full homogenization. After ultrasonic crushing at 14 *μ*m amplitude for 30 sec (Soniprep150, Sanyo, Japan), homogenate was centrifuged at 1,000xg/min for 10 min to obtain supernatant which was used to detect the levels of perixisome proliferation-activated receptor *α* (PPAR*α*), TNF-*α*, IL-1*β*, monocyte chemotactic protein-1 (MCP-1), and transforming growth factor-*β*1 (TGF-*β*1). According to the manufacturer's instructions, the above samples were measured by the corresponding ELISA kits (F15047, F15063, F11586, F15207, F16117, F16583, F16960, F15810, F16120, and F16920, Westang Biotechnology, Shanghai, China).

### 2.4. Hematoxylin-Eosin (H&E) Staining

The liver and ileum tissues of rats were fixed with 10% formalin, embedded in paraffin, and then cut into 4 *μ*m slices (EG1150C and RM2235, Leica, Germany). The slices were dewaxed with xylene, rehydrated by gradient ethanol, rinsed, stained using hematoxylin-eosin (C0105, Beyotime, Shanghai, China), dehydrated by gradient ethanol, transparent with xylene, and finally sealed in neutral balsam (G8590, Solarbio, Beijing, China). The pathological morphology of the liver and ileum tissue in each group was examined through a microscope (Olympus BX53; Olympus Corporation).

### 2.5. Oil Red O Staining and Sudan III Staining

Oil Red O stain kit (G1261, Solarbio, Beijing, China) and Sudan III stain kit (G1511, Solarbio, Beijing, China) were used to estimate the degree of hepatic steatosis in each group. The cleaned liver tissues were embedded in O.C.T. Compound (SAKURA, USA), cooled to solid state with dry ice, and then cut into 8 *μ*m sections with freezing microtome (CM1950, Leica, Germany). As specified in the manufacturer's instructions, the sections were stained and then sealed with glycerol gelatin (S2150, Solarbio, Beijing, China). Lastly, sections were imaged by means of a microscope (BX53; Olympus, Japan).

### 2.6. 16S rRNA Sequencing and Analysis

Five fresh fecal samples were taken from the intestines of each group of rats. The QIAamp fast DNA stool Mini Kit (Qiagen, Germany) was used to extract the total genomic DNA of each sample. Incorporating the barcode sequence and Illumina sequencing adapter, polymerase chain reaction (PCR) amplification was performed using universal primers (343F-5′-TACGGRAGGCAGCAG-3′, 798R-5′-AGGGTATCTAATCCT-3′), which amplified the V3-4 variable regions of bacterial 16S rRNA gene with sample DNA as the template. The amplified product was purified with Agencourt AMPure XP (Beckman Coulter, CA, USA) and sequenced on Illumina HISeq 2500 (Illumina, CA, USA) with the generation of two 250-base paired-end read cycles which were merged by FLASH (version 1.2.7). Sequences with a value of 97% similarity were clustered to the same operational taxonomy units (OTUs). Quantitative Insights into Microbial Ecology (QIIME, version 1.8.0) was the analysis tool of sequencing data that determined alpha diversity indices (chao1 metrics) and beta diversity and visualized it in principal coordinates analysis (PCoA) plots. Taxonomic analysis was performed by RDP classifier and Blast on OTUs, which was conducted through comparing RDP databases (http://rdp.cme.msu.edu/misc/resources.jsp) and Silva database (http://www.arb-silva.de) to classify the species of each OTU, and R language to visually display the species annotation results.

### 2.7. Immunohistochemistry

The ileum slices of rats were dewaxed with xylene and hydrated in gradient ethanol. The slices were treated with EDTA Antigen Retrieval Solution (P0085, Beyotime, Beijing, China) under high pressure for 20 min and 3% hydrogen peroxide for 10 min to block endogenous peroxidase. After incubation with Immunol Staining Blocking Buffer (P0102, Beyotime, Beijing, China) for 1 h, diluted primary antibody zona occludens-1 (ZO-1, 1 : 1000, ab221546, Abcam), occludin (1 : 200, ab216327, Abcam), Secretory Immunoglobulin A (sIgA, 1 : 1000, ab212330, Abcam) at 4°C for 12 h, and HRP-conjugated secondary antibodies (1 : 1000, ab97051 and ab205719, Abcam) for 1 h, the slices were treated with DAB chromogenic regent (0016, Maxim Biotechnology, Fuzhou, China) and hematoxylin, which were then observed and taken images under a fluorescence microscope (BX53; Olympus, Japan), following dehydration and seal. Protein expression was assessed by calculating protein expression score. Brown signal in the cytoplasm indicated positive staining reaction. The staining intensity was scored according to the color depth of cells in the sections, 0 point as negative, 1 point as light yellow, 2 points as yellow, and 3 points as brown. The staining range scoring was carried out based on the percentage of positive staining reaction cells to similar cells, 0 point as negative, 1 point ≤ 10%, 10% < 2 points ≤ 50%, 50% < 3 points ≤ 75%, and 4 points > 75%. The protein expression score is the product of staining intensity and staining range score.

### 2.8. Western Blot Analysis

RIPA Lysis Buffer (P0013C, Beyotime, Beijing, China) containing with PMSF (ST505, Beyotime, Beijing, China) was added into chopped ileum tissues of rats, and total proteins were extracted through homogenization, crushing, and centrifugation. The protein concentration of each sample was detected by BCA Protein Assay Kit (P0010S, Beyotime, Beijing, China) and balanced to 5 *μ*g/*μ*l by loading buffer (P0015A, Beyotime, Beijing, China). Follow the instructions of sodium dodecyl sulfate–polyacrylamide gel electrophoresis (SDS-PAGE) kit (P0012A, Beyotime, Beijing, China), 6% SDS-PAGE gels were prepared. After the protein was denaturated by boiling, 10 *μ*l protein was added to each sample well of gels, each side of which, 10 *μ*l maker (P0071, Beyotime, Beijing, China) was added as a reference, and then, electrophoresis was performed at 80 V. The protein was then transferred to PVDF membrane at 300 mA, which was sealed by 5% skimmed milk, and incubated in the primary antibody apoB48 (1 : 1000, MA5-35458, Thermo Scientific, CA, USA) and GAPDH (1 : 1000, ab181602, Abcam) at 4°C overnight. The next day, after incubation with secondary antibody of Goat anti-Rabbit (1 : 5000, ab205718, Abcam) for 2 h, membranes were developed in the chemiluminescence imaging system (Bio-Rad, CA, USA) with ECL chemiluminescence Kit (P0018S, Beyotime, Beijing, China). The expression level of target protein was relatively quantified by densitometry via ImageJ software (version 1.8.0) and comparing with the expression level of GADPH.

### 2.9. Statistical Analysis

All quantitative data were analyzed by means of SPSS software (version 22.0, IBM), and the mean ± standard deviation (SD) was used to present the data accorded with normal distribution. One-way analysis of variance (ANOVA) and Student's *t*-test were chosen to be the statistical analysis methods in this research. Value of *P* < 0.05 was considered to be statistically significant.

## 3. Results

### 3.1. Effects of SX on Liver Pathology, Liver Function, Dyslipidemia, and apoB48 Protein in NAFLD Rats

H&E staining was used to assess histopathologic changes in the liver tissue of rats after 8 weeks of HFD. As shown in Figure 2(a), the normal group had typical hepatocyte structure, clear intercellular boundaries, regular hepatic lobules, and radial hepatic cords. In the model group, there existed significant changed hepatic lobule structure, narrowed hepatic sinuses, unclear hepatic cord, and diffuse lipid accumulation around the central vein and portal vein. Under the intervention of SX, lipid changes were limited to the hepatic portal area, which presented as moderate changes in the SX-L group and slight changes in the SX-H group. In Oil Red O and Sudan III staining (Figure 2(b)), no obvious lipid droplets were found in the normal group with regular structure of hepatic sinuses and clear intercellular space. In the model group, lots of diffuse fused lipid droplets were formed, with disorganization of hepatic sinuses and hepatic cords. While lipid droplets were significantly less in the SX-H group and SX-L group which had better structure of hepatic cord and hepatic sinuses, indicating that SX can effectively prevent lipid accumulation.

As specific transaminases of the liver, AST and ALT can be increased in response to liver injury. In our results, liver function and blood lipid levels were consistent with pathological staining. Compared with the normal group, the level of ALT, AST, TC, and TG in the model group was significantly higher (*P* < 0.05, Figures 3(a)–3(d)), suggesting serious lipid deposition and liver injury in the model group. However, both low-dose and high-dose SX inhibited the elevation of ALT, AST, TC, and TG levels (*P* < 0.05), with no statistical difference from the normal group (*P* > 0.05). In addition, we also detected the expression level of PPAR*α*, a key factor in lipid metabolism, which, in the model group, was significantly lower than that in the normal group and the SX-H/L group (*P* < 0.05, Figure 3(e)), suggesting that SX might alleviate dyslipidemia by upregulating the expression of PPAR*α* to improve lipid metabolism. Moreover, the expression level of apoB48 was assessed by Western Blot. Compared with the normal group, the protein expression level of apoB48 in the model group was significantly increased, but obviously lower in the SX-H group (*P* < 0.01, Figure 3(f)), which might be relative with the increased PPAR*α* level.

### 3.2. Effects of SX on Gut Microflora Diversities in NAFLD Rats

16S rRNA sequencing and analysis was performed to investigate whether the therapeutic effect of SX was related to the changes in intestinal microbiota. The chao1 metrics shown in the violin box plot and rarefaction curves suggested that the degree of dispersion in intestinal microflora abundance distribution was higher in the model group than in the normal group, while the community richness of model was lower than the other groups (Figure 4(a)). According to the results of species annotation, it could be seen that in each group, the top five families in relative abundance of microbiota was *f_Lactobacillaceae*, *f_Prevotellaceae*, *f_Bacteroidales_S24-7*, *f_Lachnospiraceae*, and *f_Ruminococcaceae*, which all belonged to *Phylum Firmicutes* and *Bacteroidetes* (Figures 4(b) and 4(c)). Compared with the normal group, the model group decreased the relative abundance of *f_ Lactobacillaceae* and *f_Prevotellaceae* and increased *f_Bacteroidales_S24-7*, *f_Lachnospiraceae*, *f_Ruminococcaceae*, *f_Peptostrecoccaceae*, *f_Bacteroidaceae*, *f_Desulfovibrionaceae*, and *f_Erysipelotrichaceae*, while SX could upregulate the relative abundance of *f_Prevotellaceae*, and also downregulate *f_Bacteroidales_S24-7*, *f_Lachnospiraceae*, *f_Ruminococcaceae*, *f_Erysipelotrichaceae*, and *f_Desulfovibrionaceae* (Figure 4(b)). In the PCoA diagram, the closer the sample distance between each group is, the smaller the difference in the microbial composition would be. Based on the results of taxonomic analysis, there were a long distance in the PCoA diagram and less consistency in the heat map between the model group and the normal group, indicating a significant difference in the microbial composition of two groups (Figures 5(a) and 5(b)). Yet closer distance existed between the normal group and the SX-H/L group, as well as higher consistency in the heat map, suggesting that the normal group and the SX-H/L group had similar microbial composition (Figures 5(a) and 5(b)). In conclusion, the intervention of SX could regulate the relative abundance in the gut microbiota of NAFLD rats and make it tending to normal.

### 3.3. Effects of SX on Gut Barrier Function in NAFLD Rats

H&E staining was used to evaluate the intestinal mucosal injury. The results showed that intestinal mucosa in the normal group rats had clear and complete tissue structure, thick and continuous muscle layers, and orderly arranged cells without pathological changes of edema or congestion, while the intestinal mucosal of the model group presented necrotic epithelial cells, widened villous space, missing or disorganized crypts (Figure 6(a)). The intervention of SX reduced the intestinal mucosal injury to varying degrees, and the effect of the SX-L group was more obvious (Figure 6(a)). To evaluate the integrity of the intestinal barrier, we performed immunohistochemistry to detect the expression level of tight junction proteins in ileal mucosa, consisting of ZO-1, occludin, and sIgA. As is shown by our results, in the model group, the expression levels of ZO-1 and occludin were significantly decreased, but sIgA were significantly increased (*P* < 0.05, *P* < 0.01; Figures 6(b) and 6(c)), suggesting intestinal barrier hypofunction. The expression levels of ZO-1 and occludin, however, in SX-H/L group, were significantly higher, and sIgA was significantly lower than those in the model group (*P* < 0.05, Figures 6(b) and 6(c)), which had no difference in protein expression from the normal group (*P* > 0.05, Figures 6(b) and 6(c)), reflecting normal intestinal barrier function.

### 3.4. Effects of SX on Inflammatory Level in NAFLD Rats

The level of plasma LPS was examined by ELISA and was significantly higher in the model group than in the normal group (*P* < 0.05, Figure 7(a)), while treatment with high-dose or low dose SX made LPS level nearly drop to normal (*P* > 0.05). Besides, the levels of proinflammatory factors IL-1*β* and TNF-*α*, chemokine MCP-1, and fibrosis-related factor TGF-*β* were significantly increased in the model group but decreased in the SX-H/L group (*P* < 0.05, Figures 7(b)–7(e)), manifesting that SX can mitigate inflammation of NAFLD rats by downregulating the levels of LPS, IL-1*β*, TNF-*α*, MCP-1, and TGF-*β*1.

## 4. Discussion

The lipid deposition, liver function, and blood fat levels in HFD-fed rats appeared obvious improvement under the intervention of SX, consistent with our previous research which did not discuss the impact of SX on lipoproteins expression, intestinal microbiota, and liver inflammation [31]. In this research, the significant amelioration of SX on NAFLD rats was concerned with the expression of apoB48 and PPAR*α*, the regulation of gut microbiota, and intestinal barrier function.

We found that SX could increase the level of PPAR*α* as well as reduce the expression of apoB48. In the intestinal epithelial cells, apoB48 is assembled with microsomal triglyceride transfer protein (MTP), TG, cholesteryl ester (CE), and other particles to form mature TG-rich lipoproteins, CMs, and VLDL, which enter the blood circulation through the lacteals and the mesenteric lymphatic duct and of which remnants is absorbed by the liver after being ingested by adipocytes and myocytes [32]. Mager et al. found that the elevation time of apoB48 after meal in NAFLD children was prolonged, suggesting accumulation of CMs remnants [33]. It was reported that matoa fruit peel could decrease liver lipid content, TG level, visceral fat, and body weight and may play the antiobesity role in HFD-fed rats by inhibiting the secretion of apoB48 to reduce intestinal lipid absorption [34]. Similarly, in our results, the decrease of apoB48 expression was consistent with blood fat levels and liver lipid deposition. In fact, excess lipids would be discharged from the liver through VLDL, which meant the decrease of VLDL-containing apoB48 secreted by the liver could cause the relative increase of liver TG with the decrease of serum TG [35]. Our results suggested that SX might also work by inhibiting the absorption of intestinal lipids to reduce the production of CMs, rather than restraining the secretion of VLDL-containing apoB48 from the liver. Fatty acid consumption is mainly achieved in liver mitochondria by fatty acid *β*-oxidation which is a strategy to control liver lipid accumulation and obesity [36]. PPAR*α* mainly modulates the intake of lipids and the *β*-oxidation of peroxisomes [37, 38]. The loss of PPAR*α* decreased fatty acid *β*-oxidation and aggravated hepatic steatosis in mice [9]. We analyzed the level of PPAR*α* in the liver of each group and found that PPAR*α* in the model group was significantly lower than that in the normal group. By promoting the expression of PPAR*α*, the expression of fatty acid *β*-oxidation genes can be stimulated, while inflammation and oxidative stress genes are inhibited, as well as lipid *β*-oxidation and bile acid excretion are accelerated, thus promoting lipid metabolism. [39, 40]. Studies have reported that PPAR*α*-mediated increased catabolism of fatty acids played a protective role in NAFLD and NASH [41]. In our results, SX-H intervention led to upregulation of PPAR*α* in NAFLD rats, possibly through the *β*-oxidation pathway to increase fatty acid decomposition and reduce lipid accumulation. It was found that the lack of PPAR*α* could lead to the increase of the secretion and serum level of apoB48, while the activator of PPAR*α* inhibited the expression of apoB48R mRNA [42, 43]. Our results also showed a negative correlation between PPAR*α* and apoB48, suggesting that the decreased expression of apoB48 might be due to the increase of the PPAR*α* level.

There is growing evidence of a strong link between gut microbiota and NAFLD [44]. This study showed that SX could effectively regulate the relative abundance of intestinal microbiota and was similar to that of the normal group. Analysis of species composition changes showed that *f_Prevotellaceae* decreased in the model group, while SX reversed this change. Recent studies have shown that *Prevotella/Bacteroidetes* ratio predicts weight and fat loss after a 24-week dietary intervention [45]. In addition, *Prevotella* was mainly involved in carbohydrate and monosaccharide metabolism and can produce short-chain fatty acids (SCFA) which are beneficial to intestinal health [46]. The *f_Lachnospiraceae* family is a phylogenetic and morphologically heterogeneous taxa belonging to firmicutes, which can produce SCFA, convert primary bile acids to secondary bile acids, and promote resistance to intestinal pathogen colonization [46, 47]. However, some studies have suggested that the high abundance of *f_Lachnospiraceae* was positively correlated with glucose and lipid metabolism indicating metabolic disorders [48]. Our results were consistent with Zeng et al.'s finding that HFD-fed mice had a higher abundance of *f_Lachnospiraceae* than mice fed a low-fat diet [49]. Otherwise, SX could reduce the relative abundance of *f_Desulfovibrionaceae* and *f_Erysipelotrichaceae* caused by NAFLD. *Desulfovibrio* belongs to *Proteobacteria*, which is a sulfate reducing bacterium and can produce H_2_S, positively correlated with the level of LPS [50]. Recent studies shown that the increase of IgA content may be related to the disorder of intestinal microbiota, and the level of sIgA in our model group also represented an upward tendency, which is probably caused by the excessive growth of pathogenic microorganism in intestine immune response [51]. In the intestinal lumen, IgA binds and “wraps” disease-causing pathogens and prevents infection through neutralization and rejection [52]. In intestinal disease, the *f_Erysipelotrichaceae* family belonging to *Firmicutes* was found to be highly IgA coated [53]. In fact, *f_Erysipelotrichaceae* could produce palmitic, stearic, oleic and fatty acids, which might lead to metabolic disturbances, stimulate the production of proinflammatory cytokines and enhance the response of T-helper cells [53]. Therefore, the alleviation of lipid disorder and intestinal inflammation by SX might also be related to the downregulation of *f_Erysipelotrichaceae* abundance. *B. subtilis and E. faecium* from *Firmicutes* had been studied to change the abundance of intestinal flora in NAFLD, promote beneficial bacteria, and inhibit harmful bacteria, as well as upregulate the expression of PPAR*α* protein [22]. SX not only improved the abundance of gut microbiota but also promoted the expression of PPAR*α*, showing a connection between lipid metabolic proteins and the abundance of intestinal microbiota.

The integrity of intestinal barrier is related to the homeostasis of gut microbiota which is manifested in the disruption of the intestinal mucosal barrier when intestinal microbiota is disturbed [22]. Tight junction proteins, ZO-1 and occludin, play an important role in maintaining the monolayer integrity of intestinal epithelial cells [54]. ZO-1 is a cytoplasmic plaque protein that connects transmembrane protein and cytoskeleton, while occludin can affect the tight junction of intestinal epithelial cells by regulating macromolecular flux, both of which are indicator of mucosal integrity, and decreased expression indicates impaired barrier integrity [55, 56]. In our results, the expression of ZO-1 and occludin in the intestinal tract of NAFLD rats was significantly reduced but increased after SX intervention, suggesting that SX could repair the intestinal barrier by increasing the expression of ZO-1 and occludin, which was consistent with the above conclusion. Incomplete intestinal mucosa impairs the function of intestinal barrier, presenting as the “leaky gut” that permits bacterial toxic metabolites such as LPS to leak from the intestinal lumen into the systemic circulation and eventually reach the liver [57]. As a natural ligand of Toll-like receptor 4 (TLR4), LPS stimulates an inflammatory signaling cascade through the LPS-TLR4-NF-*κ*B/PI3K axis, resulting the release of many proinflammatory cytokines, such as TNF-*α*, IL-1*β*, and IL-18 [58]. Similarly, in our results, LPS, TNF-*α*, IL-1*β*, MCP-1, and TGF-*β*1 were elevated along with the barrier integrity impairment, suggesting the formation of “leaky gut” in NAFLD. Nevertheless, the intervention of SX downregulated the level of LPS, TNF-*α*, IL-1*β*, MCP-1, and TGF-*β*1 by repairing mucosal integrity to recovery the intestinal barrier function.

In conclusion, our study confirmed that the gut-liver axis was one of the possible ways for SX to improve NAFLD, that is, to regulate the expression of apoB48 and PPAR*α* and protect the intestinal barrier function by changing the relative abundance of gut microbiota, thus reducing the lipid deposition and inflammatory response in the liver. Otherwise, our study suggested that there was a certain correlation between lipid metabolic proteins and the abundance of intestinal microbiota, however, between which specific regulatory pathway still needed to be confirmed by further research.

## Figures and Tables

**Figure 1:** SX ameliorated NAFLD rats induced by HFD via the gut-liver axis. SX: Shugan Xiaozhi decoction; NAFLD: nonalcoholic fatty liver disease; HFD: high-fat diet; FFAs: free fatty acids; TC: total cholesterol; TG: triglyceride; apoB48: apolipoprotein B48; CMs: chylomicrons; PPAR*α*: peroxisome proliferator activated receptor *α*; LPS: lipopolysaccharide; sIgA: secretory immunoglobulin A; ZO-1: zona occludens 1.

**Figure 2:** SX alleviated hepatic steatosis in HFD-induced NAFLD rats. (a) H&E staining shown that liver steatosis was ameliorated by the treatment of SX (200x magnification). (b) Oil red O and Sudan III staining indicated that SX inhibited lipid accumulation in the liver of NAFLD rats (400x magnification).

**Figure 3:** SX promoted lipid metabolism by raising hepatic PPAR*α* level and reducing the expression of intestinal apoB48. (a–e) The level of ALT, AST, TC, TG, and PPAR*α* were improved by SX treatment. (f) The protein expression level of apoB48 treated with SX was decreased in plasma of NAFLD rats. Values are represented as mean ± SD (*n* = 10). ^∗^*P* < 0.05, ^∗∗^*P* < 0.01 vs. the normal group; ^#^*P* < 0.05, ^##^*P* < 0.01 vs. the HFD-induced model group.

**Figure 4:** Effect of SX on the gut microbiota in NAFLD rats. (a) Community richness analysis based on chao1 metrics. (b) Relative abundance of microbiota at phylum level. (c) Relative abundance of microbiota at family level. Group A: model group; Group B: normal group; Group G: SX-L group; Group H: SX-H group.

**Figure 5:** SX could regulate gut microbiota diversities in NAFLD rats. (a) Heat map of community structure differences and cluster analysis at family level. (b) Graph of PCoA between the different groups. Group A (A01-A05): model group; Group B (B01-B05): normal group; Group G (G01-G05): SX-L group; Group H (H01-H05): SX-H group.

**Figure 6:** SX could protect intestinal mucosal and barrier integrity on NAFLD rats. (a) H&E staining indicated that intestinal mucosal treated with SX was protected from HFD-induced damage (100x magnification). (b, c) The expression level of ZO-1, occludin, and sIgA manifested that SX improved the intestinal barrier function on NAFLD rats (200x magnification). Values are represented as mean ± SD (*n* = 10). ^∗^*P* < 0.05, ^∗∗^*P* < 0.01 vs. the normal group; ^#^*P* < 0.05, ^##^*P* < 0.01 vs. the HFD-induced model group.

**Figure 7:** SX alleviated inflammation in HFD-induced NAFLD rats. (a–e) The level of LPS, TNF-*α*, IL-1*β*, MCP-1, and TGF-*β*1 were reversed by SX treatment. Values are represented as mean ± SD (*n* = 10). ^∗^*P* < 0.05, ^∗∗^*P* < 0.01 vs. the normal group; ^#^*P* < 0.05, ^##^*P* < 0.01 vs. the HFD-induced model group.

## Data Availability

The datasets used and/or analyzed during the current study are available from the corresponding author on reasonable request.
